The article "circ_0062491 alleviates periodontitis via the miR-142-5p/IGF1 axis" was retracted in 2023. Reasons: duplicated images; concerns about the images; concerns about a third party's involvement.

# circ_0062491 alleviates periodontitis via the miR-142-5p/IGF1 axis

**DOI:** 10.1515/med-2022-0442

**Published:** 2022-04-08

**Authors:** Chunlin Wang, Junxia Gong, Dai Li, Xianghui Xing

**Affiliations:** Department of Pediatric Dentistry, Nanjing Stomatological Hospital, Medical School of Nanjing University, Xuanwu District, Nanjing, Jiangsu 210000, China; Department of First Outpatient, Nanjing Stomatological Hospital, Medical School of Nanjing University, Nanjing, China

**Keywords:** periodontitis, periodontal ligament stem cells, circ_0062491, osteogenic differentiation, miR-142-5p, *IGF1*

## Abstract

CircularRNAs (circRNAs) are collectively involved in periodontitis. The aim of this study was to explore the roles of circ_0062491 in osteogenic differentiation of PDLSCs and provide a novel method for periodontitis treatment. mRNA and protein expression levels were measured by qRT-PCR and western blotting. Alkaline phosphatase (ALP) and alizarin red S (ARS) staining were used to detect the activity of osteogenesis. Furthermore, the interactions between miR-142-5p and circ_0062491/*IGF1* were verified by a luciferase reporter assay. circ_0062491 was suppressed in PDL tissues of periodontitis patients and overexpressed in osteogenesis-induced PDLSCs. Upregulated circ_0062491 promoted osteogenic differentiation of PDLSCs. miR-142-5p was verified to be a target of circ_0062491, and the overexpression of miR-142-5p suppressed the osteogenic differentiation of PDLSCs induced by circ_0062491 Additionally, miR-142-5p targeted *IGF1,* and silenced *IGF1* abrogated the effects of suppressed miR-142-5p on osteogenic differentiation of PDLSCs. In conclusion, circ_0062491 acted as a competing endogenous RNA to regulate osteogenic differentiation of PDLSCs via the miR-142-5p/*IGF1* axis.

## 1 Introduction

Periodontitis is a common inflammatory disease with oral pathogenic microorganisms as the initiating factor and periodontal pocket formation and alveolar bone resorption as the main clinical features [1,2]. Under the stimulation of periodontal pathogenic bacteria, a large number of inflammatory factors are accumulated in the periodontal tissue to activate the inflammatory response process and break the homeostasis of bone remodeling, resulting in the decrease of the body’s osteogenic ability and the damage of periodontal bone tissue [3,4]. For example, Isola et al. [5] reported that NLRP3 inflammasome was a promising biomarker of disease risk in patients with periodontitis. Matarese et al. [6] demonstrated that transglutaminase 2 was involved in molecular mechanisms of inflammatory response occurring in periodontal disease. These research studies implied that inflammation was a key in periodontitis. Therefore, the study of the inflammation pathogenesis of periodontitis is of great significance for the prevention and treatment of the disease.

Periodontal ligament stem cells (PDLSCs) are adult stem cells existing in periodontal tissues, which have high biological properties of proliferation, clone formation, self-renewal, and multiple differentiation [7]. When subjected to diseases or external stimulation, PDLSCs can promote tissue regeneration through continuous proliferation and targeted differentiation [8,9]. Interestingly, periodontitis is an inflammatory response dominated by the local immune response, which invades and destroys the periodontal tissue, leading to the loss of the regeneration ability of the periodontal tissue [3]. Therefore, the study on the differentiation ability of PDLSCs is helpful to further explore the pathological mechanisms of periodontitis.

Circular RNAs (circRNAs) are a subset of noncoding RNAs (ncRNAs) that have recently been emerged as new regulators of gene expression [10,11,12]. Recently, it has become common to verify circRNAs by demonstrating that they are resistant to degradation by ribonuclease R (RNase R) [13]. The helicase activity of RNase R can degrade highly structured RNAs, including ribosomal RNAs. The exonic and intronic of the circular RNAs would be enriched after RNase R treatment, while linear RNAs would be consumed [14,15]. Meanwhile, as one of the largest gene families, miRNAs are ncRNAs with a length of about 19–24 nucleic acids, which are widely found in eukaryotic cells [16]. CircRNAs act as miRNA sponges and competitively inhibit transcriptional regulation of miRNAs to function as a new type of competing endogenous RNA (ceRNA) regulator [17,18]. CircRNAs can bind or release a large number of miRNAs more quickly and stably, and play its role in regulating miRNA efficiently; furthermore, ceRNA activity of circRNAs is more prominent than linear ceRNA [10,11,12]. CircRNAs have been reported to be good biomarkers in various diseases including periodontitis [19,20,21]. circ_0062491 is a novel circRNA in periodontitis identified by sequencing technology combined with experimental validation [22]; however, the underlying molecular mechanisms of circ_0062491 in PDLSCs remain to be further investigated.

Therefore, according to the previous study, we further investigated the molecular mechanisms of circ_0062491 in the development of periodontitis. Furthermore, we hypothesized that circ_0062491 sponges miR-142-5p to regulate insulin-like growth factor I (*IGF1)* expression to regulate osteogenic differentiation of PDLSCs. Additionally, four clinicians were involved in all stages of the study.

## 2 Materials and methods

### 2.1 Periodontal ligament (PDL) tissue

Periodontitis patients diagnosed at Nanjing Stomatological Hospital from 1 January 2020 to 1 January 2021 were obtained (sex: 24 males, 16 females; age: 31 ± 3 years old; periodontal pocket depth: 5.45 ± 0.78 mm; bleeding on probing (%): 39.15 ± 11.36), as well as healthy volunteers (sex: 17 males, 23 females; age: 31 ± 3 year old). All subjects have provided informed consent. Inflammatory PDL tissues (*n* = 40) were obtained from periodontitis patients with no systemic diseases (*n* = 40), whereas healthy PDL tissues (*n* = 40) were obtained from teeth extracted for an orthodontic reason. In simple terms, the teeth were rinsed with sterile PBS, and the tissues were gently separated from the middle part of the root surface. Some tissues were used to detect RNA levels, while the rest were used to isolate PDLSCs. The clinical research about the collection of periodontal ligament tissues has been approved by the Ethics Committee of Nanjing Stomatological Hospital (No. NSC20190926012) in accordance with the declaration of Helsinki.

### 2.2 Cell culture

The PDL tissues were minced into small pieces and treated with collagenase type I (1 mg/mL; Sigma-Aldrich, NJ, USA) digestion under 37°C for 0.25 h. Then, cell suspensions were filtered and cultured in DMEM (Gibco, CA, USA) containing 10% FBS (Gibco, CA, USA), 2 mM L-glutamine (Gibco, CA, USA), and 1% penicillin/streptomycin (Gibco, CA, USA). After 14 days of incubation, the cells were digested and single-cell derived colony cultures were obtained using the limiting dilution technique. PDLSCs were obtained through dilution and passed 5 times.

### 2.3 Cell transfection

Overexpressed circ_0062491 vector (circ_0062491), downregulated circ_0062491 (si-circ_0062491 1#, si-circ_0062491 2#), overexpressed miR-142-5p negative control (nc mimic), overexpressed miR-142-5p (mimic), suppressed miR-142-5p negative control (nc inhibitor), suppressed miR-142-5p (inhibitor), and downregulated IGF1 (si-IGF1 1#, si-IGF1 2#) in this study were all bought from GenePharma (Shanghai, China). PDLSCs were cultured at a concentration of 2 × 10^5^ cells per well in six-well plates. After the cells had grown to about 50% confluence, corresponding plasmids were transfected into PDLSCs using Lipofectamine 3000 reagent (Life Technologies, CA, USA), with all procedures following the manufacturer’s protocol.

### 2.4 Osteogenic differentiation

PDLSCs from periodontitis patients reaching 80% confluence in 6-well plates were incubated with osteogenic medium (100 nM dexamethasone, 50 mg/mL ascorbic acid, and 5 mM b-glycerophosphate; Sigma-Aldrich, NJ, USA) for 7 or 14 days, and the medium was changed every 3 days. The alkaline phosphatase (ALP) activity assay was performed after 7 days of incubation with osteogenic medium using an ALP kit according to the instruction manual (Jiancheng, Nanjing, China). For ALP staining, an ALP Staining Kit (Beyotime, Nantong, China) was used after the cells were washed with distilled water three times. The positive PDLSCs were photographed by a microscope (Zeiss, Oberkochen, Germany), and observed at 562 nm on an absorbance microplate reader (BioTek, Winooski, USA) to quantify ALP staining activity. Alizarin red S (ARS) staining was performed after 14 days of incubation with an osteogenic medium. After the cell culture medium was discarded, PDLSCs were washed twice with PBS. Then, PDLSCs were fixed with 10% formaldehyde buffer for 10 min and then rinsed with distilled water 3 times. Afterward, 0.1% alizarin red-tris-HCl dye solution (pH 8.3) was added and stained at 37°C for 0.5 h. After rinsing with distilled water, the positive cells were observed at an absorbance of 405 nm (BioTek, Winooski, USA). All experiments were repeated three times.

### 2.5 Stability of circRNA

Actinomycin D (2 mg/mL; Sigma-Aldrich, NJ, USA) and RNase R (Epicentre, WI, USA) were used to test the stability of circ_0062491; the stability was measured by quantitative real-time polymerase chain reaction (qRT-PCR).

### 2.6 Ribonuclease R (RNase R) treatment

RNase R treatment is mainly used for circRNA identification and enrichment experiments [23]. About 10 μg of total RNA, which was extracted as previously described in the qRT-PCR section, was treated with 20 mg/mL RNase R (Genesee, Guangzhou, China) at 37°C for 1 h, followed by RNase R inactivation at 65°C for 20 min and a control group without RNase R treatment was set. RNA was then extracted using a miRNeasy Mini Kit (QIAGEN, Dusseldorf, Germany) and washed with distilled water. Reverse transcription was performed using the SuperScript First-Strand Synthesis Kit (Invitrogen, Calif, USA) and random primers (Invitrogen, CA, USA) following the manufacturer’s standard protocol.

### 2.7 qRT-PCR

Total RNA of PDL tissues as well as PDLSCs of each group was extracted using TRIzol reagent (Invitrogen, CA, USA) and converted into cDNA (SuperScript First-Strand Synthesis Kit; Invitrogen, CA, USA). GAPDH was used as housekeeping control for circ_0062491 and mRNAs. U6 was used as an internal reference for miR-142-5p. Primer sequences for circ_0062491, miR-142-5p, and all mRNAs were designed by RiboBio (Guangzhou, China). qRT-PCR was performed using the SYBR Green Premix Ex TaqTM kit (Takara, Kusatsu, Japan) and the Applied Biosystems 7500 Real-Time PCR Detection System. The data were analyzed using the 2^−ΔΔCt^ relative expression method. All experiments were repeated three times.

### 2.8 Western blotting assay

Osteogenic differentiation-related proteins including osteocalcin (OCN), runt-related transcription factor 2 (RUNX2), and collagen type I alpha1 (COL-1) were measured in PDLSCs. Total protein was extracted from PDLSCs by lysis in RIPA buffer. Protein concentrations were determined with the BCA kit (Sigma-Aldrich, NJ, USA). Additionally, proteins were isolated using 12% SDS-PAGE gel and were moved onto PVDF membranes (Bio-rad, CA, USA). The membranes were blocked with 5% milk for 2 h and then incubated with primary antibodies for one night at 4°C. Immune complexes were incubated with horseradish peroxidase-conjugated anti-rabbit or anti-mouse IgG antibodies (Abcam, CA, USA). Finally, protein expressions were captured using the Western-Light Chemiluminescent Detection System (Peiqing, Shanghai, China). All experiments were repeated three times. Primary antibodies were purchased from Abcam (CA, USA): anti-OCN (1/1,000, ab133612), anti-RUNX2 (1/1,000, ab236639), anti-COL-1 (1/1,000, ab34710), and GADPH (1/1,000, ab8245).

### 2.9 Dual luciferase reporter assay

The wild-type circ_0062491 or IGF1 3′-UTR, mutant-type circ_0062491 or IGF1 3′-UTR were synthesized and cloned into pmirGLO luciferase vectors (Promega, Madison, USA) to determine whether miR-142-5p directly targets circ_0062491 or the IGF1. The miR-142-5p mimic negative control plasmids (nc mimic), miR-142-5p mimic (mimic), and Renilla luciferase plasmid (Promega, Madison, USA) were co-transfected into PDLSCs. Firefly and Renilla luciferase activities were measured consecutively by a Dual-Luciferase Reporter Assay kit (K801-200; BioVision Tech, San Francisco, USA).

### 2.10 Statistical analysis

Data were analyzed with GraphPad Prism version 8.3 (GraphPad Software, CA, USA), and presented as mean ± SD. Student’s *t*-test (two groups) and one-way ANOVA (multiple groups) were applied for difference analysis. *p* value < 0.05 was deemed statistically significant.

## 3 Results

### 3.1 circ_0062491 was suppressed in periodontitis patients, and positively related to PDLSC osteogenic differentiation

The circ_0062491 expression level was significantly decreased in PDL tissues of periodontitis patients compared with the normal group (Figure 1a). The incubation time of PDLSCs in the osteogenic medium was proportional to the expression of circ_0062491 and peaked on day 14 (Figure 1b). Then, the results of RNase R treatment indicated that the expression level of linear 0062491 was substantially decreased compared with circ_0062491 (Figure 1c). Furthermore, the half-life period of circ_0062491 was more than 24 h while the half-life period of its linear form was less than 4 h (Figure 1d).

**Figure 1:** Expression levels of circ_0062491 in periodontitis tissues and cells. (a) The expression of circ_0062491 in PDL tissues was measured by qRT-PCR. (b) The expression of circ_0062491 in PDLSCs was determined by qRT-PCR. (c) qRT-PCR analysis for the expression of circ_0062491 and lnc_0062491 in PDLSCs after RNaseR treatment. (d) qRT-PCR analysis for the expression of circ_0062491 and lnc_0062491 in PDLSCs at the indicated time after treatment with actinomycin D. *p < 0.05, **p < 0.01, ***p < 0.001. vs healthy, control, mock, and circular group.

### 3.2 Overexpressed circ_0062491 promoted osteogenic differentiation of PDLSCs

As shown in Figure 2a, the expression of circ_0062491 was significantly increased after transfection in PDLSCs. The number and activity of ALP positive cells as well as ARS positive cells were increased by upregulated circ_0062491 (Figure 2b), so did the mRNA and protein expression levels of OCN, RUNX2, and COL-1 (Figure 2c and d).

**Figure 2:** Overexpressed circ_0062491 promoted osteogenic differentiation of PDLSCs. (a) circ_0062491 expression levels were detected by qRT-PCR in PDLSCs after transfection. (b) Images and quantification of ALP staining and ARS of PDLSCs transfected with circ_0062491. (c) qRT-PCR analysis for the expression of OCN, RUNX2, and COL-1. (d) Western blotting analysis for the expression of OCN, RUNX2, and COL-1. **p < 0.01, vs the vector group.

### 3.3 circ_0062491 targeted miR-142-5p in PDLSCs

The binding sites between circ_0062491 and miR-142-5p were predicted with the online database Starbase3.0 (Figure 3a). Dual luciferase assay further indicated that overexpressed miR-142-5p dramatically decreased the luciferase activity of PDLSCs transfected with wild-type 3′-UTR of circ_0062491, whereas this phenomenon was not observed in the mutant-type group (Figure 3b). Then, overexpression of circ_0062491 decreased the expression level of miR-142-5p in PDLSCs (Figure 3c). Furthermore, miR-142-5p was markedly upregulated in PDL tissues of periodontitis patients compared with healthy controls while it was suppressed in osteogenic differentiation PDLSCs over time up to 21 days cultured in the osteogenic medium (Figure 3d and e).

**Figure 3:** circ_0062491 targeted miR-142-5p in PDLSCs. (a) Bioinformatics predicted the binding sites between miR-142-5p and circ_0062491. (b) Dual-luciferase reporter assay confirmed that miR-142-5p was a target of circ_0062491 in PDLSCs. (c–e) qRT-PCR analysis was performed to detect the expression of miR-142-5p in PDL tissues and PDLSCs. *p < 0.05, **p < 0.01, ***p < 0.001. vs nc mimic, vector, healthy and control group.

### 3.4 Overexpression of miR-142-5p reversed the effects of circ_0062491 on osteogenic differentiation of PDLSCs

Subsequently, in order to further explore the relationship between miR-142-5p and circ_0062491, we performed a rescue experiment. The cells were co-transfected with circ_0062491 and miR-142-5p mimic. The expression of miR-142-5p was remarkably downregulated by the miR-142-5p inhibitor and upregulated by miR-142-5p mimic, suggesting that PDLSCs were successfully transfected (Figure 4a). Upregulation of ALP and ARS activity (Figure 4b) as well as mRNA and protein expression levels of OCN, RUNX2, and COL-1 induced by circ_0062491 were obviously reversed by overexpressed miR-142-5p (Figure 4b–d).

**Figure 4:** Overexpression of miR-142-5p reversed the effects of circ_0062491 on osteogenic differentiation of PDLSCs. (a) miR-142-5p expression levels were detected by qRT-PCR. (b) Images and quantification of ALP staining and ARS of PDLSCs transfected with circ_0062491 and miR-142-5p mimic. (c) qRT-PCR analysis for the expression of OCN, RUNX2, and COL-1. (d) Western blotting analysis for the expression of OCN, RUNX2, and COL-1. **p < 0.01, vs nc inhibitor and control group. #*p* < 0.05, ##*p* < 0.01, vs nc mimic and circ_0062491 + nc mimic group.

### 3.5 miR-142-5p directly targeted *IGF1* in PDLSCs.

TargetScan 7.2 predicted the binding sites between *IGF1* and miR-142-5p (Figure 5a). Dual luciferase assay further confirmed the interaction between *IGF1* and miR-142-5p (Figure 5b). The mRNA expression of *IGF1* was significantly increased by circ_0062491 and suppressed by a miR-142-5p mimic in PDLSCs (Figure 5c). Additionally, *IGF1* was remarkably downregulated in the PDL tissue of periodontitis patients, and significantly upregulated in osteogenic differentiation PDLSCs over time up to 21 days cultured in the osteogenic medium (Figure 5d and e).

**Figure 5:** *IGF1* was the target gene of miR-142-5p. (a) Bioinformatics predicted the binding sites between miR-142-5p and *IGF1*. (b) Dual-periodontitis luciferase reporter assay was conducted to confirm the association between *IGF1* and miR-142-5p. (c–e) The expression of *IGF1* was determined by qRT-PCR. *p < 0.05, **p < 0.01, ***p < 0.001. vs nc mimic, vector, healthy and control group. ##*p* < 0.01, vs nc mimic group.

### 3.6 Silenced *IGF1* inhibited the effects of downregulated miR-142-5p

As shown in Figure 6a, *IGF1* expression was significantly decreased after the interference RNA of *IGF1* was transfected into PDLSCs, which was more potent in the si-IGF1 2# group (Figure 6a). Furthermore, APL and ARS activities as well as expression levels of OCN, RUNX2, and COL-1 were markedly increased by suppressed miR-142-5p; however, downregulated *IGF1* then abrogated these effects of the miR-142-5p inhibitor on PDLSCs (Figure 6b–d).

**Figure 6:** Effects of *IGF1* on PDLSCs. (a) *IGF1* expression levels were detected by qRT-PCR. (b) Images and quantification of ALP staining and ARS of PDLSCs transfected with miR-142-5p inhibitor and si-IGF1. (c) qRT-PCR analysis for the expression of OCN, RUNX2, and COL-1. (d) Western blotting analysis for the expression of OCN, RUNX2, and COL-1. *p < 0.05, **p < 0.01, vs si-nc, and control group. #*p* < 0.05, ##*p* < 0.01, vs inhibitor + si-nc group.

## 4 Discussion

In the present study, circ_0062491 was suppressed in the PDL tissue of periodontitis patients, and overexpressed circ_0062491 promoted osteogenic differentiation of PDLSCs, which is one of the key factors for periodontitis. Additionally, circ_0062491 sponged miR-142-5p to promote the downregulation of *IGF1*. Together, we unveiled the underlying mechanisms that circ_0062491 promoted the osteogenic differentiation of PDLSCs derived from periodontitis patients via regulating the miR-142-5p/IGF1 axis, which is also shown in graphical abstract.

The current clinical treatment for periodontitis mainly includes basic and surgical treatment, but these methods still cannot completely repair the damaged periodontal tissue [24]. Recently, the research on early biomarkers of periodontitis has become a new hotspot. Many studies have demonstrated that metalloproteinase-8, macrophage inflammatory protein-1 alpha, interleukin-1 beta, interleukin-6, and hemoglobin, and their combinations were promising host-derived biomarkers for early diagnosis of periodontitis [25]. Besides, circRNAs were demonstrated to be novel biomarkers for the diagnosis of periodontitis, such as circular RNA CDR1as [20], circular RNA 0081572 [26], and so on. This study demonstrated that circ_0062491 was decreased in periodontitis, indicating that circ_0062491 might also be a potential biomarker for periodontitis.

In recent years, PDLSCs have been reported to play an important role in the clinical application of periodontal tissue repair and regeneration [7]. Many transcription factors and signaling pathways are involved in the osteogenic differentiation of PDLSCs, including circRNAs with relatively stable structures and functions [19,27].

Gu et al. found 1456 circRNAs with abnormal expression in PDLSCs from osteogenic induction culture compared with the normal culture group through RNA sequencing. KEGG database analysis results indicated that these circRNAs may be involved in the osteogenic differentiation of stem cells [28]. Li et al. found that circRNA CDR1 acted as a sponge for miR-7 and regulates the upregulation of growth differentiation factor 5 and the phosphorylation of Smad1/5/8 and P38 MAPK, thereby promoting the osteogenic differentiation of PDLSCs [20]. Wang et al. found that the circRNA expression level also changed during the osteogenic differentiation of PDLSCs induced by mechanical force [29]. These studies confirm that circRNA may play an important regulatory role in the osteogenesis of PDLSCs.

circ_0062491 was identified to be aberrantly expressed in PDL tissues [22] and was found to be suppressed in PDL tissues derived from patients with periodontitis in this study. Furthermore, the expression of circ_0062491 increased with the time of osteogenesis induction of PDLSCs. Next, overexpressed circ_0062491 promoted the secretion of bone matrix mineralization and osteogenic differentiation-associated proteins, indicating that circ_0062491 may be a potential biomarker of osteogenic differentiation in PDLSCs.

Then, miR-142-5p was verified to be a target miRNA of circ_0062491 and was upregulated in PDL tissues and suppressed in osteogenesis-induced PDLSCs. In a study examining the effects of alcohol on the inflammatory phase of fracture healing, miRNA microarray analysis of callus tissues suggested significant upregulation of miR-142-5p [30]. In addition, Wei et al. found that miR-142-5p was also significantly upregulated during the differentiation of mouse preosteoblasts into mature osteoblasts (0 to 21 days) [31]. These findings suggest that miR-142-5p may be involved in the regulation of osteogenic differentiation and maintenance of osteoblast activity during fracture healing. However, the effects of miR-142-5p on osteogenic differentiation of PDLSCs have not yet been reported. Our data suggested that overexpression of miR-142-5p reversed the effects of circ_0062491 on osteogenic differentiation of PDLSCs.

IGF-1 is closely related to tooth development and the differentiation of odontogenic stem cells and can promote the proliferation and differentiation of odontoblasts and PDLSCs [32,33]. In this research, IGF-1 was confirmed to be a target gene of miR-142-5p and suppressed in PDL tissues, and upregulated in osteogenesis-induced PDLSCs. Furthermore, suppressed IGF-1 alleviated the effects of suppressed miR-142-5p on osteogenic differentiation of PDLSCs.

However, this study has some limitations. For instance, only 40 samples of periodontitis were obtained in this study. Therefore, we need to collect more samples to make our conclusions more accurate and reliable. Further studies are needed to focus on the regulation of circ_0062491 in periodontitis *in vivo*.

## 5 Conclusion

This research demonstrated that circ_0062491 was decreased in periodontitis. Overexpressed circ_0062491 promoted osteogenic differentiation of PDLSCs. Additionally, our findings suggested that circ_0062491 acted as a ceRNA to regulate osteogenic differentiation of PDLSCs via the miR-142-5p/*IGF1* axis. Overexpression of circ_0062491 may be an alternative for the treatment of periodontitis.
